# The Combination of ^18^F-Fluorodeoxyglucose Positron Emission Tomography Metabolic and Clinical Parameters Can Effectively Distinguish Rheumatoid Arthritis and Polymyalgia Rheumatic

**DOI:** 10.1155/2022/9614678

**Published:** 2022-04-11

**Authors:** Guanyun Wang, Xiaofei Liu, Jiaxin Chen, Fengyan Zhang, Xiaodan Xu, Yanmei Wang, Ruimin Wang, Shulin Yao, Jian Zhu, Zhiwei Guan

**Affiliations:** ^1^Department of Nuclear Medicine, The First Medical Center, Chinese PLA General Hospital, 28 Fuxing Road, Haidian District, Beijing, China; ^2^Nuclear Medicine Department, Beijing Friendship Hospital, Affiliated to Capital Medical University, Beijing, China; ^3^Department of Rheumatology and Immunology, Hainan Hospital, Chinese PLA General Hospital, 80 Jianglin Road, HaiTang District, Sanya, Hainan, China; ^4^Medical School of Chinese PLA, Fuxing Road 28, Beijing, China; ^5^Department of Rheumatology and Immunology, The First Medical Center, Chinese PLA General Hospital, 28 Fuxing Road, Haidian District, Beijing, China; ^6^GE Healthcare China, Pudong New Town, Shanghai, China

## Abstract

**Objective:**

To evaluate ^18^F-fluorodeoxyglucose positron emission tomography (^18^FDG PET) and clinical parameters to differentiate rheumatoid arthritis (RA) and polymyalgia rheumatic (PMR). *Patients and Methods*. This retrospective study evaluated 54 patients with suspected RA (*n* = 23) and PMR (*n* = 31) who underwent ^18^F-FDG PET/CT before treatment. The complete diagnosis was based on each classification criterion and at least followed up for 6 months. Demographic and clinical data were also collected. Semiquantitative analysis (maximum standardized uptake value, SUVmax) of abnormal ^18^F-FDG uptake was undertaken at 17 musculoskeletal sites, and two scoring systems (mean reference (liver/control) scores) were evaluated. The differential diagnostic efficacy of each independent parameter was evaluated using the receiver operating characteristic (ROC) curve. Integrated discriminatory improvement (IDI) and bootstrap tests were used to evaluate the improvement in diagnostic efficacy using a combination of multiple parameters.

**Results:**

The ROC curve analysis of SUVmax indicated that the interspinous ligament showed the highest discriminative diagnostic value (sensitivity, 64.5%; specificity, 78.3%; area under the curve (AUC), 0.764; positive predictive value, 0.800; negative predictive value, 0.621). The combined model with the rheumatoid factor (RF) and metabolic parameters of ^18^F-FDG PET resulted in the highest AUC of 0.892 and showed significant reclassification by IDI (IDI, 9.51%; 95% confidence interval: 0.021–0.175; *P* = 0.013). According to the bootstrap test, compared with RF alone, the combination of RF and metabolic parameters showed an improvement in ROC and was statistically significant (*P* = 0.017).

**Conclusions:**

The combination of ^18^F-FDG PET metabolic and clinical parameters can further improve the differential diagnosis of RA and PMR.

## 1. Introduction

Rheumatoid arthritis (RA) is also one of the most prevalent chronic inflammatory autoimmune diseases and is characterized by painful swollen joints [1, 2]. Polymyalgia rheumatic (PMR) is a chronic, common, unexplained systemic inflammatory disease that affects people aged ≥50 years [3, 4]. PMR is characterized by pain and long-term morning stiffness affecting the neck, shoulders, hips, upper arms, and thighs and is frequently accompanied by cranial and large vessel subtypes of giant cell arteritis (GCA) [3, 4]. Due to RA and PMR being different in major goals of treatments, the early diagnosis for the patient is necessary. PMR is not erosive and does not cause structural damage. However, RA can cause cartilage and bone damage as well as disability. Thus, for RA patients, early diagnosis is key to optimal therapeutic success, particularly in patients with well-characterized risk factors for poor outcomes such as high disease activity, presence of autoantibodies, and early joint damage [2]. Remarkably, patients experiencing RA need to preserve their joint and muscular function at an early stage and are only partially responsive to low doses of prednisone [5]. In the clinic, the diagnosis of RA and PMR is usually based on the pattern of symptoms, physical examination, serologic testing results (such as rheumatoid factor (RF) and anti-cyclic citrullinated peptide antibody (anti-CCP Ab)), and imaging findings [1, 4, 6]. Therefore, it is difficult to differentiate PMR from RA in clinical practice.

^18^F-fluorodeoxyglucose positron emission tomography (^18^FDG PET) can be applied aggressively to detect inflammatory disorders [7]. ^18^FDG PET has been proven to play a role in the diagnosis of RA and PMR, especially in evaluating the physical status of patients [8–10]. However, in the differential diagnosis of RA and PMR, the role of ^18^FDG PET is still controversial due to the lack of research data.

The main aim of this study is to assess the diagnostic utility in discriminating RA from PMR and to assess the additional diagnostic value of ^18^FDG PET to clinical parameters.

## 2. Patients and Methods

### 2.1. Patients

From January 2014 to July 2021, we retrospectively identified patients with suspected RA and PMR who underwent ^18^F-FDG PET/CT before treatment from our hospital database. Patients with RA were diagnosed according to the 2010 ACR/EULAR classification criteria for RA [11], and patients with PMR were diagnosed according to the 2012 European League Against Rheumatism (EULAR) and the American College of Rheumatology (ACR) classification criteria [12]. All RA and PMR patients were followed for at least 6 months. Besides, we collected the patients who were without rheumatic disease or malignancy from January 2014 to July 2021 and were assigned to the control group. All included patients were aged ≥50 years and had complete data on demographics, clinical, and laboratory tests.

Demographic, clinical, and laboratory data were also collected. Baseline laboratory tests included blood examination, C-reactive protein (CRP), erythrocyte sedimentation rate, immunoglobulin G, RF, anti-keratin antibody (AKA), anti-CCP Ab, and anti-neutrophil cytoplasmic antibodies (ANCA).

This is a retrospective cohort study, and all patients were informed and signed before ^18^F-FDG PET/CT. According to current China national guidelines, this study did not require ethical approval.

### 2.2. PET/CT Scanning

All patients were scanned using ^18^F-FDG PET/CT (Biograph 64, GE Healthcare). Patients fasted for 4−6 h with plasma glucose levels <11.1 mmol/L and rested for at least 20 min in a quiet waiting room before intravenous administration of ^18^F-FDG (^18^F-FDG; Atomic High-Tech Co., Ltd., radiochemical purity of >95%) at 3-4 MBq/kg. The low-dose CT (LDCT) parameters were voltage = 120 kV, current = 100 mAs, rotation = 0.8, layer thickness = 5 mm, and pitch = 1. The parameters of PET included 3-dimensional mode, 2.5 min/bed (30% overlap), 4-5 beds/person, three iterations, 21 subsets, Gaussian filter half-height width = 4.0 mm. PET/CT scan was performed after 45−60 min, beginning from the skull base to the upper femur in free-breathing mode, with a 3 min emission scan/bed and CT attenuation correction.

### 2.3. Image Analysis

A multiparametric analysis prototype (Siemens, Germany), a dedicated prototype postprocessing tool, was used for the imaging analysis. A total of 17 musculoskeletal sites were specifically assessed (two acromioclavicular joints, two periarticular shoulder regions, two sternoclavicular joints, two sacroiliac joints, two hip joints, two greater trochanter bursas, two symphysis pubis entheses, two ischial tuberosities, and most PET-avid interspinous ligaments). Large vessels were also evaluated for abnormal maximum standardized uptake value (SUVmax) ≥2, consistent with concomitant GCA [13].

Quantitative analyses were performed by two experienced nuclear medicine physicians (WGY and GZW) blinded to the clinical information of the patients. The qualitative analysis comprised a visual evaluation of ^18^F-FDG uptake using the following scoring system: 0, no uptake (same as bone); 1, lower than normal liver uptake; 2, similar to normal liver uptake; and 3, higher than normal liver uptake [14].

For semiquantitative analysis, a region of interest was drawn around each site, and the SUVmax was calculated in the RA, PMR, and control groups. The average SUVmax for each measurement site in the RA and PMR groups was measured and divided by the control group from the same measurement site to calculate the score for the semiquantitative scoring system. The semiquantitative scoring system was as follows: 0, lower than the control group; 1, similar to the control group; 2, higher than the control group, but not more than twice; and 3, higher than twice or more.

### 2.4. Statistical Analysis

All data were analyzed using the *R* software (version 4.0.2; Bell Laboratories, USA). Continuous variables are presented as mean ± standard deviation, and categorical variables are presented as percentages. The distribution of baseline characteristics and PET multiple parameters among the three groups (RA, PMR, and controls) were analyzed using the Mann−Whitney *U* test, chi-square test, or variance analysis. The optimal cutoff values of the baseline characteristics and PET parameters for differential diagnosis were determined using receiver operating characteristic (ROC) analyses. Diagnostic accuracy parameters including sensitivity, specificity, positive predictive value, and negative predictive value were evaluated. Logistic regression was used to select the most efficient parameter for the combined model in the differential diagnosis. The integrated discriminatory improvement (IDI) from the *PredictABEL* package and the bootstrap test from the *pROC* package were calculated for the comparison of diagnostic models. Differences were considered statistically significant at *P* < 0.05.

## 3. Results

### 3.1. Demographics, Clinical, and Laboratory Characteristics

A total of 54 patients were included in this retrospective analysis, including 23 with RA patients (42.6%) and 31 patients with PMR (57.4%). Additionally, a total of 50 control participants were included in the study.

Table 1 compares the baseline characteristics between the RA and PMR groups and the control group, and the clinical parameters between RA and PMR. The results showed no differences in sex and age between the three groups. Meanwhile, white blood cell count (WBC, 7.3 ± 2.9 vs. 15.9 ± 27.7, *P* = 0.046), CRP (3.6 ± 5.0 vs. 5.5 ± 5.4, *P* = 0.049), RF positive (60.9% vs. 3.2%, *P* < 0.001), AKA positive (43.5% vs. 0.0%, *P* < 0.001), anti-CCP Ab positive (65.2% vs. 6.5%, *P* < 0.001), and ANCA positive (52.2% vs. 16.1%., *P* = 0.007) were statistically different between RA and PMR.

### 3.2. ^18^F-FDG PET

All patients with PMR showed nonabnormal vascular ^18^F-FDG uptake without large vessel GCA. SUVmax, mean reference (liver) score, and mean reference (control) score for each site and were compared between the RA and PMR groups (Table 2).

SUVmax for interspinous ligament (1.8 ± 0.8 vs. 2.8 ± 1.2, *P* = 0.001), sacroiliac joint (1.8 ± 0.5 vs. 2.3 ± 0.9, *P* = 0.010), hip joint (1.8 ± 0.6 vs. 2.8 ± 2.0, *P* = 0.040), trochanter (1.8 ± 0.8 vs. 2.3 ± 0.9, *P* = 0.006), and ischial tubercle (1.6 ± 0.9 vs. 2.5 ± 1.2, *P* = 0.002) were significantly lower in patients with RA than that in patients with PMR.

The degree of ^18^F-FDG uptake as measured by mean reference score compared with normal liver and SUVmax in RA was significantly lower in cases than in PMR only in the ischial tubercle (1.0 ± 1.0 vs. 1.7 ± 1.0, *P* = 0.024). The degree of ^18^F-FDG uptake as measured by mean reference score compared with the control group and SUVmax in the RA group was significantly lower than that in the PMR group in the interspinous ligament (0.8 ± 1.0 vs. 1.6 ± 0.8, *P* = 0.003), sacroiliac joint (0.8 ± 1.0 vs. 1.4 ± 0.9, *P* = 0.037), trochanter (0.5 ± 0.8vs. 1.1 ± 1.0, *P* = 0.020), symphysis pubis (1.2 ± 1.0 vs. 1.7 ± 0.6, *P* = 0.038), and ischial tubercle (0.8 ± 1.0 vs. 1.6 ± 0.8, *P* = 0.003).

Overall, these results indicate that the SUVmax, mean reference (liver) scores, and mean reference (control) scores for some sites (ischial tubercle, interspinous ligament, sacroiliac joint, etc.) can distinguish between the RA and PMR groups.

### 3.3. Sensitivity and Specificity of ^18^F-FDG PET Findings for Differential Diagnosis of RA and PMR

Table 3 summarizes the results for the best-performing musculoskeletal sites based on the ROC analysis. The ROC analysis of SUVmax indicated that the interspinous ligament showed the highest discriminative diagnostic value with a sensitivity of 64.5%, specificity of 78.3%, area under the curve (AUC) of 0.764 (*P* = 0.001), positive predictive value (PPV) of 0.800, and negative predictive value (NPV) of 0.621. Logistic regression analyses of the total ^18^F-FDG PET metabolic parameters showed that sensitivity was 90.3%, specificity was 78.3%, AUC was 0.832 (*P* < 0.001), PPV was 0.800, and NPV was 0.842.

The ROC analysis of the degree of ^18^F-FDG uptake measured by mean reference score compared with the control group and SUVmax indicated that the ischial tubercle showed the highest discriminative diagnostic value with a sensitivity of 64.5%, specificity of 78.3%, AUC of 0.764 (*P* = 0.001), PPV = 0.722, and NPV = 0.722. The combination based on the logistic regression with all sites showed a sensitivity of 90.3%, specificity of 60.9%, AUC of 0.757 (*P* < 0.001), PPV of 0.757, and NPV of 0.824. Regarding clinical parameters, RF and anti-CCP Abs, both achieved high sensitivity (96.8%; 93.5%) and moderate specificity (60.9%; 65.2%) values for differential diagnosis. The combined model with RF and SUVmax of ^18^F-FDG PET resulted in the highest AUC of 0.892. The models are presented below.

(1) $$\begin{array}{c} y=\frac{1}{1+e^{-\left(0.75\times \text{interspinous ligament}+0.52\times \text{sacroiliac joint}+0.35\times \text{hip joint}-0.25\times \text{trochanter}+0.40\times \text{ischial tubercle}-3.54\times \text{RF}-2.68\right)}}. \end{array}$$

The diagnostic efficiencies of the three models that combined the clinical and metabolic parameters of ^18^F-FDG PET are shown in Figure 1. All accuracy analyses were based on cross-validation. Finally, according to the analyses of IDI in Table 4, the combination of RF and ^18^F-FDG PET metabolic parameters allowed a significant reclassification with IDI of 9.51% (95% confidence interval, 0.021–0.175; *P* = 0.013), and according to the bootstrap test, compared with RF alone, the combination of RF and metabolic parameters of ^18^F-FDG PET had a statistically significant improvement in ROC (*D* = 2.309; boot: *n* = 2000; boot: stratified = 1; *P* = 0.017). Both indicated statistical diagnostic benefits with multiparametric combination in the differential diagnosis of RA and PMR.

## 4. Discussion

The most important result of our study was that between the three methods, the measurement of musculoskeletal site SUVmax was the most valuable for the differential diagnosis between RA and PMR, and the proportion of patients with RA with abnormal SUVmax at five sites, including the interspinous ligament, sacroiliac joint, hip joint, trochanter, and ischial tubercle, were significantly lower than those of patients with PMR. Moreover, we compared SUVmax or clinical parameters only, and the combination of abnormal ^18^F-FDG uptake and clinical parameters was sufficiently discriminated between the two groups.

Due to differences in treatment and prognosis, it is important to distinguish between RA and PMR at an early stage. In the clinic, the differential diagnosis of RA and PMR has always been difficult, especially with elderly onset rheumatoid arthritis (EORA) [15]. The functional prognosis and treatment response are different in patients with RA and PMR [16]. Therefore, the successful identification of RA and PMR is essential. Laboratory tests for RA-related autoantibodies RF and ACPA, including AKA and anti-CCP Abs, may help in the differential diagnosis of RA and PMR. However, laboratory tests show normal (seronegative) in approximately one-third of patients with RA [2]. Conventional imaging modalities, such as ultrasound, have been shown to play an important role in the diagnosis of RA and PMR, and the new 2012 EULAR/ACR clinical classification criteria are the most commonly used criteria for the classification of rheumatic polymyalgia in clinics, which has high sensitivity [12, 17]. However, the new 2012 EULAR/ACR classification criteria for polymyalgia rheumatica with the use of ultrasound showed different results in discriminating PMR from RA [12, 18].

In recent years, the use of ^18^F-FDG PET/CT to evaluate inflammatory conditions, including arthritis and rheumatic disease, has been increasingly reported, and ^18^F-FDG PET/CT has certain clinical value in the therapeutic monitoring and follow-up of RA and PMR [7, 10]. Some studies have shown that ^18^F-FDG PET/CT also has a certain value in the differential diagnosis of RA and PMR, especially EORA. Yamashita et al. found that according to PET/CT findings, ischial tuberosity, greater trochanters, and spinous processes could help discriminate between RA and PMR [19]. Takahashi et al. examined the differential diagnosis of PMR from EORA and showed that a high sensitivity (92.6%) and specificity (90.0%) were obtained if three of the following five items were positive, including uptake in the ischial tuberosity and spinous process, absence of uptake at the wrist, linear or circular uptake around the shoulders, and isolated uptake of the iliopectineal bursa [20]. Another study also showed that ^18^F-FDG PET/CT is useful to differentiate PMR from EORA. Abnormal FDG accumulation was observed in patients with PMR in the entheses, suggesting the presence of enthesitis in addition to bursitis and synovitis [15]. In our study, we selected patients with RA aged ≥50 years, which can be matched to the age of patients with PMR. We found that SUVmax could better distinguish between RA and PMR than the other two scores. SUVmax in five musculoskeletal sites showed significant differences between the two groups. Similar to the above studies, it was suggested that FDG uptake could distinguish between RA and PMR. We also demonstrated that the combination of high uptake at these sites of the musculoskeletal system provided high specificity (90.3%) and moderate specificity (69.6%) in the differential diagnosis of RA and PMR.

However, relying solely on FDG could not yet achieve a good differential diagnosis ability, which is similar to the diagnostic ability of common clinical parameters, such as RF and anti-CCP. Therefore, we combined ^18^F-FDG PET metabolic parameters with clinical parameters, and the differential diagnosis ability was improved compared with a single diagnostic pattern. Through IDI and bootstrap tests, we found that the combination of ^18^F-FDG PET metabolic parameters and RF can increase diagnostic ability compared with RF alone. This diagnostic model not only maintains high sensitivity but also has higher specificity.

This study had some limitations. First, this was a retrospective study involving a small number of patients, which could bias the statistics and diagnostic model. Second, in this study, PET/CT scans only included the trunk, and limb bones and facets were not included in the study. Third, the control group established by collecting normal people did not obtain better results. It depends mainly on SUVmax, which may be cumbersome for the diagnosis of diseases. Therefore, large-scale and prospective multicenter studies should be performed to improve future research and establish a more recommended and effective diagnostic model through more research.

## 5. Conclusions

In conclusion, clinical parameters and ^18^F-FDG PET showed varying diagnostic efficacy in the differentiation of RA and PMR. The combination of ^18^F-FDG PET metabolic and clinical parameters could further improve the differential diagnosis.

## Figures and Tables

**Figure 1:** The ROC curves of the combination of SUVmax (AUC = 0.832), RF (AUC = 0.788), and the combined model (the combination of SUVmax plus RF, AUC = 0.892).

**Table 1:** The differences in demographics between rheumatoid arthritis (RA), polymyalgia rheumatic (PMR), and control, and clinical parameters between RA and PMR.

Characteristic	RA (*n* = 23)	PMR (*n* = 31)	Control (*n* = 50)	*P* value
Demographics				
Age	65.8 ± 8.5	68.8 ± 9.5	68.7 ± 9.9	0.530^*∗*^
Male (*n*%)	13 (56.5%)	12 (38.7%)	20 (40.0%)	0.345^*∗*^
Clinical parameters				
HGB (g/L)	111.0 ± 23.1	103.6 ± 17.7	—	0.248
WBC (10^9^/L)	7.3 ± 2.9	15.9 ± 27.7	—	**0.046**
PLT (10^9^/L)	274.2 ± 115.1	317.9 ± 96.6	—	0.091
NEUT (10^9^/L)	0.7 ± 0.1	0.9 ± 0.8	—	0.411
LYM (10^9^/L)	0.2 ± 0.1	0.5 ± 1.3	—	0.972
CRP (mg/dL)	3.6 ± 5.0	5.5 ± 5.4	—	**0.049**
ESR (mm/h)	49.4 ± 37.0	61.7 ± 29.6	—	0.132
IGG (mg/dl)	1403.6 ± 610.5	1400.7 ± 340.0	—	0.733
RF positive (*n*%)	14 (60.9%)	1 (3.2%)	—	<**0.001**
AKA positive (*n*%)	10 (43.5%)	0 (0.0%)	—	<**0.001**
anti-CCP Ab positive (*n*%)	15 (65.2%)	2 (6.5%)	—	<**0.001**
ANCA positive (*n*%)	12 (52.2%)	5 (16.1%)	—	**0.007**

^*∗*^Variance analysis. HGB: hemoglobin; WBC: white blood cell; PLT: platelet; NEUT: neutrophil; LYM: lymphocyte; CRP: C-reactive protein; ESR: erythrocyte sedimentation rate; IgG: immunoglobulin G; RF: rheumatoid factor; AKA: anti-keratin antibody; anti-CCP Ab: anti-cyclic citrullinated peptide antibody; ANCA: anti-neutrophil cytoplasmic antibodies. The significance of bold values is *P* < 0.05, which means differences were considered statistically significant.

**Table 2:** The SUVmax and qualitative scores (mean reference score compared to normal liver and mean reference score compared to the control group) for cases compared with controls at each musculoskeletal site.

Musculoskeletal site	RA	PMR	*P* value
SUVmax			
Acromioclavicular joint	2.1 ± 1.3	2.3 ± 1.1	0.180
Shoulder	2.7 ± 1.4	3.9 ± 2.5	0.076
Sternoclavicular joint	2.3 ± 1.6	2.2 ± 0.9	0.489
Interspinous ligament	1.8 ± 0.8	2.8 ± 1.2	**0.001**
Sacroiliac joint	1.8 ± 0.5	2.3 ± 0.9	**0.010**
Hip joint	1.8 ± 0.6	2.8 ± 2.0	**0.040**
Trochanter	1.8 ± 0.8	2.3 ± 0.9	**0.006**
Symphysis pubis	2.2 ± 2.3	2.1 ± 0.9	0.080
Ischial tubercle	1.6 ± 0.9	2.5 ± 1.2	**0.002**

Mean ref. (liver) score cases			
Acromioclavicular joint	1.4 ± 1.2	1.4 ± 1.0	0.902
Shoulder	2.1 ± 1.0	2.0 ± 1.0	0.804
Sternoclavicular joint	1.7 ± 0.9	1.4 ± 0.9	0.445
Interspinous ligament	1.4 ± 0.7	1.8 ± 1.0	0.092
Sacroiliac joint	1.4 ± 0.7	1.6 ± 0.8	0.339
Hip joint	1.4 ± 0.9	1.6 ± 1.0	0.508
Trochanter	1.3 ± 0.9	1.6 ± 1.0	0.166
Symphysis pubis	1.2 ± 0.8	1.4 ± 0.8	0.313
Ischial tubercle	1.0 ± 1.0	1.7 ± 1.0	**0.024**

Mean ref. (control) score cases			
Acromioclavicular joint	0.9 ± 1.0	1.3 ± 0.9	0.158
Shoulder	1.1 ± 1.0	1.5 ± 0.9	0.117
Sternoclavicular joint	1.2 ± 0.9	1.5 ± 0.9	0.134
Interspinous ligament	0.8 ± 1.0	1.6 ± 0.8	**0.003**
Sacroiliac joint	0.8 ± 1.0	1.4 ± 0.9	**0.037**
Hip joint	1.3 ± 1.0	1.6 ± 0.8	0.221
Trochanter	0.5 ± 0.8	1.1 ± 1.0	**0.020**
Symphysis pubis	1.2 ± 1.0	1.7 ± 0.6	**0.038**
Ischial tubercle	0.8 ± 1.0	1.6 ± 0.8	**0.003**

RA: rheumatoid arthritis; PMR: polymyalgia rheumatic; SUV max: maximum standardized uptake value. The significance of bold values is *P* < 0.05, which means differences were considered statistically significant.

**Table 3:** Differential diagnostic efficiency of SUVmax and qualitative scores (mean reference score compared to control) and clinical parameters with receiver operating characteristic analysis.

Variable	AUC	*P* value	Sen (%)	Spe (%)	PPV	NPV
SUVmax						
Interspinous ligament	0.764	0.001	64.5	78.3	0.800	0.621
Sacroiliac joint	0.705	0.010	48.4	82.6	0.789	0.542
Hip joint	0.664	0.041	51.6	82.6	0.800	0.559
Trochanter	0.718	0.007	71.0	65.2	0.733	0.625
Ischial tubercle	0.753	0.002	83.9	56.5	0.722	0.722
Combination	0.832	<0.001	90.3	69.6	0.800	0.842

Mean ref. (control) score cases						
Interspinous ligament	0.712	0.008	83.9	56.5	0.722	0.722
Sacroiliac joint	0.658	0.048	67.7	60.9	0.700	0.583
Trochanter	0.663	0.042	51.6	82.6	0.800	0.559
Symphysis pubis	0.671	0.033	90.3	34.8	0.651	0.727
Ischial tubercle	0.730	0.004	83.9	56.5	0.722	0.722
Combination	0.794	<0.001	90.3	60.9	0.757	0.824

Clinical parameters						
RF positive	0.788	<0.001	96.8	60.9	0.769	0.933
AKA positive	0.717	0.007	100.0	43.5	1.000	0.705
anti-CCP Ab positive	0.794	<0.001	93.5	65.2	0.784	0.882

AUC: area under curve; SUV max: maximum standardized uptake value; Sen: sensitivity; Spe: specificity; PPV: positive predictive value; NPV: negative predictive value; RF: rheumatoid factor; anti-CCP Ab: anti-cyclic citrullinated peptide antibody.

**Table 4:** Comparison of the combination with ^18^F-FDG PET metabolic parameters and clinical parameters to only clinical parameters with IDI.

Variable	AUC	Sen (%)	Spe (%)	*P* value	IDI (%)	95% CI	*P* value
Combination1	0.892	90.3	82.6	**<0.001**	9.51	0.015–0.176	**0.021**
Combination2	0.884	93.5	73.9	**<0.001**	7.79	0.003–0.153	**0.041**
Combination3	0.882	93.5	73.9	**<0.001**	—	—	—

Combination1: the combination of SUVmax plus RF; Combination2: the combination of SUVmax plus anti-CCP Ab; Combination3: the combination of SUVmax plus RF plus anti-CCP Ab; AUC: area under curve; SUVmax: maximum standardized uptake value; Sen: sensitivity; Spe: specificity; IDI: integrated discrimination improvement; 95% CI: 95% confidence interval. The significance of bold values is *P* < 0.05, which means differences were considered statistically significant.

## Data Availability

The data used to support the findings of this study are available from the first author upon reasonable request.
